The article "Plasmablastic Lymphoma: A Review of Current Knowledge and Future Directions" was retracted in 2016. Reasons: plagiarized text; overlap with other authors' work.

# Plasmablastic Lymphoma: A Review of Current Knowledge and Future Directions

**DOI:** 10.1155/2015/315289

**Published:** 2015-08-18

**Authors:** Ghaleb Elyamany, Eman Al Mussaed, Ali Matar Alzahrani

**Affiliations:** ^1^Department of Pathology and Blood Bank, Prince Sultan Military Medical City, P.O. Box 7897, Riyadh 11159, Saudi Arabia; ^2^Department of Hematology, Theodor Bilharz Research Institute, Egypt; ^3^Hematopathology Division, Department of Basic Science, College of Medicine, Princess Nourah Bint Abdulrahman University, Riyadh, Saudi Arabia; ^4^Department of Oncology, Prince Sultan Military Medical City, Saudi Arabia

## Abstract

Plasmablastic lymphoma (PBL) is an aggressive subtype of non-Hodgkin's lymphoma (NHL), which frequently arises in the oral cavity of human immunodeficiency virus (HIV) infected patients. PBL shows diffuse proliferation of large neoplastic cells resembling B-immunoblasts/plasmablasts, or with plasmacytic features and an immunophenotype of plasma cells. PBL remains a diagnostic challenge due to its peculiar morphology and an immunohistochemical profile similar to plasma cell myeloma (PCM). PBL is also a therapeutic challenge with a clinical course characterized by a high rate of relapse and death. There is no standard chemotherapy protocol for treatment of PBL. Cyclophosphamide, doxorubicin, vincristine, and prednisone (CHOP) or CHOP-like regimens have been the backbone while more intensive regimens such as cyclophosphamide, vincristine, doxorubicin, high-dose methotrexate/ifosfamide, etoposide, high-dose cytarabine (CODOX-M/IVAC), or dose-adjusted etoposide, prednisone, vincristine, cyclophosphamide, and doxorubicin (DA-EPOCH) are possible options. Recently, a few studies have reported the potential value of the proteasome inhibitor bortezomib and thalidomide in PBL patients. The introduction of genes encoding artificial receptors called chimeric antigen receptors (CARs) and CAR-modified T cells targeted to the B cell-specific CD19 antigen have demonstrated promising results in multiple early clinical trials. The aim of this paper is to review the recent advances in epidemiology; pathophysiology; clinical, pathologic, and molecular characteristics; therapy; and outcome in patients with PBL.

## 1. **Introduction**

Plasmablastic lymphoma (PBL) is a rare lymphoma associated with immunosuppression. It is strongly associated with human immunodeficiency virus (HIV) infection and often occurs within the oral cavity. PBL is also seen in elderly patients with age-associated immunosuppression and other patients receiving immunosuppressive therapy; however, despite its predisposition for the immunocompromised patients, PBL has been diagnosed in immunocompetent patients [1, 2].

The article "Plasmablastic Lymphoma: A Review of Current Knowledge and Future Directions" was retracted in 2016. Reasons: plagiarized text; overlap with other authors' work.

This lymphoma is now considered a separate diagnostic entity, distinct from diffuse large B-cell lymphoma (DLBCL), not otherwise specified, in the 2008 World Health Organization (WHO) classification of lymphoid neoplasms [3].

HIV-related lymphomas are frequently associated with EBV. Dual infection with EBV and human herpesvirus 8 (HHV8) has been demonstrated in PBL [4]. Cases of PBL occurring in immunocompetent patients have been documented and increasingly described particularly in HIV-negative patients [5–7].

Since the initial reports of PBL [1], it has been described in several other sites, including the gastrointestinal tract, omentum, lung, nasal and paranasal regions, testes, bones, soft tissue, lymph nodes, bone marrow, skin, and CNS [8–13]. PBL has also been documented to arise from long-standing sacrococcygeal cysts in HIV-positive persons [14].

Although the clinical and pathologic features of this lymphoma are well characterized, its molecular pathogenesis remains poorly understood, partly owing to its rarity [15, 16].

The diagnosis of PBL remains a diagnostic challenge given its rarity, peculiar morphology, and an immunohistochemical profile similar to PCM. Additionally, there is a wide differential diagnosis within the subgroup of DLBCL and PCM with plasmablastic morphology that is still a common problem because of the lack of a distinctive phenotype [17]. Distinction between extramedullary plasmablastic neoplasms remains critical for patient management, and correlation with clinical findings is essential [18].

Currently, very little is known about the molecular characteristics of PBL. Array comparative genomic hybridization (aCGH) involving 16 PBLs demonstrated that the genomic aberration pattern of PBL is more similar to DLBCL than to PCM [19], despite the high degree of immunophenotypical similarity between PBL and PCM [20].

The clinical course of PBL is characteristically aggressive. It is generally associated with early dissemination and poor response to therapy and has a reported median overall survival (OS) time of 15 months [16]. Currently, treatment responses are usually partial and temporary; however, prolonged and durable responses to chemotherapy [14, 21, 22] have been reported.

The main goal of this paper is to systematically review the most recent advances in epidemiology; pathophysiology; clinical, pathologic, and molecular characteristics; therapy; and prognosis in patients with PBL.

## 2. Epidemiology

PBL is primarily a disease of adults, affecting men more often than women. The M/F ratio is 5.7 : 1 for the oral type and 4 : 1 for the extraoral type [15]. It is strongly associated with HIV infection and, in the setting of HIV infection, the most frequent site of involvement is the oral cavity. It can also affect other extranodal sites with a predilection for mucosal tissues.

The article "Plasmablastic Lymphoma: A Review of Current Knowledge and Future Directions" was retracted in 2016. Reasons: plagiarized text; overlap with other authors' work.

PBL has also been reported in HIV-negative persons, particularly those who have immunosuppression. In the last decade, several case reports and series have been published, accounting for 590 cases [23]. PBL involving extraoral sites have been reported in several immunocompetent individuals [24–30].

PBL is a rare entity, thought to account for approximately 2.6% of all AIDS-related lymphomas (ARLs) [31, 32]. It is unclear if the actual incidence of PBL has increased in recent years. The apparent increase in published case reports and series could be a reflection of an increased awareness of PBL among clinicians and pathologists [33]. Furthermore, the actual incidence of PBL not associated with HIV infection has not yet been determined. In a literature review of 228 patients with PBL, 157 patients (69%) were HIV-positive and 71 (31%) were HIV-negative [26]; among HIV-negative patients, 33% of the patients have some form of immunosuppression, most often solid organ transplantation or steroid therapy [15]. The remainder of the HIV-negative patients are apparently immunocompetent. In a recent case series from Korea, none of the patients reported showed evidence of immunosuppression [28].

The majority of patients with PBL are middle-aged adults with a mean age at presentation of 39 years in HIV-positive patients and 58 years in HIV-negative patients [16]. Although the majority of patients are adults, PBL has also been reported in the pediatric age group [24, 34–40]; however, a literature review identified only 17 cases. It is unclear if there is a racial or ethnic predominance in PBL patients. However, cases have been reported in populations from different continents [6]. The median age was 10 years (range 2–17), >80% with advanced stage at presentation and jaw/oral cavity as the most common site of initial disease [41]; however, extranodal locations have also been reported. Prognosis is usually poor, with two reported long-term survivors [41, 42].

The actual prevalence of human herpesvirus 8 (HHV8) infection in PBL is more controversial, possibly depending on the sensitivity of the techniques used. On the basis of available literature HHV8 testing was reported in 27 out of 68 cases, and results were positive in only 4 (14.81%) [43].

## 3. Pathogenesis

The pathogenesis of PBL is poorly understood and likely determined by the complexity of biological interplays between HIV-related immunodeficiency, molecular events, coinfecting oncogenic viruses, and chronic immune activation [33].

The article "Plasmablastic Lymphoma: A Review of Current Knowledge and Future Directions" was retracted in 2016. Reasons: plagiarized text; overlap with other authors' work.

It has been proposed that ARLs may develop along four pathogenetic pathways involving EBV and HHV8 infection, as well as c-MYC, p53, and BCL-6 gene aberrations [44].

The contribution of HIV to PBL pathogenesis might develop through four main mechanisms, the duration and the degree of immunodeficiency or immunosuppression; chronic B-cell proliferation/exhaustion due to chronic antigenic stimulation; loss of immune control of oncogenic herpesvirus as EBV; and an incomplete immune reconstitution or factors unrelated to immune dysfunction [45–50]. Similar to other ARLs, such as Burkitt lymphoma (BL) and immunoblastic and primary effusion lymphoma (PEL), PBL has a strong association with Epstein-Barr virus (EBV) infection, and EBV infection is associated with prevention of apoptosis in B-cells by several mechanisms related to EBV antigens [23, 24].

In HIV-associated PBL, 74% of the cases showed the presence of EBV within the tumor cells [16]. EBV infection has been demonstrated based on the expression of EBV-encoded RNA (EBER) [26]. The association between PBL and HHV8 at this time is unclear.

It has been proposed that Kaposi sarcoma-associated HHV8 may play a relevant role in the pathogenesis of PBL. A few studies have demonstrated expression of HHV8-associated proteins in PBL [51, 52]; however, other studies do not support such an association [30, 53]. Furthermore, it is unclear if these HHV8-associated PBL cases originated from multicentric Castleman disease, which should place them in a different category [54].

Based on immunohistochemical, molecular, and genetic studies, PBL probably develops from postgerminal center, terminally differentiated, active B-cells in transition from immunoblasts to plasma cells [23]. In these processes, there are chromosomal aberrations likely associated with the development of malignancy. A recent study has shown recurring rearrangements involving* MYC* and the immunoglobulin gene [55];* MYC* gene rearrangements involving the *κ* and *λ* light chain genes and other non-Ig genes have also been described [23]; however, it is not sufficient to cause lymphoma, because low levels of t(8; 14)(q24; q32) have been detected in healthy individuals by using highly sensitive polymerase chain reaction [56]. It has been suggested that aberration of the genes involved in cell cycle regulation may contribute to PBL oncogenesis. Hypermethylation of the* p16* gene has been reported [57], and* MYC* upregulation by translocation between the* MYC* gene and immunoglobulin heavy chain gene (*MYC*/*IgH*) was reported recently in 3 separate case reports [58].

## 4. Clinical Features

PBL is characterized for its predilection of involving the oral cavity of HIV-positive individuals as originally described [1]. Following the first report, a number of cases have been reported in extraoral sites, in HIV-positive cases. The most commonly affected sites are the GI tract, lymph nodes, and skin [11, 16]. A similar pattern is seen in patients with HIV-negative PBL, with the oral cavity and GI tract being the most commonly involved sites [39].

The article "Plasmablastic Lymphoma: A Review of Current Knowledge and Future Directions" was retracted in 2016. Reasons: plagiarized text; overlap with other authors' work.

The frequency of oral involvement is higher in HIV-positive (58%) than in HIV-negative patients (16%) [26]. Other less common extraoral sites include the CNS [59, 60], paranasal sinus [27, 60], mediastinum, lungs [8, 27, 61], liver [61], and testes [11]. Bone marrow involvement has been reported at 30% in both HIV-positive and HIV-negative patients [26].

No significant differences in age and gender have been reported between oral and extraoral PBL. The peak of incidence for the oral and extraoral types occurs at 41 years (range 7–86 years) and 46 years (range 11–86 years), respectively, and both are more common in males [15].

In both HIV-positive and HIV-negative patients, most present with rapid growing, sometimes destructive, disease in advanced clinical stage (Ann Arbor stage 3 or 4), with elevated LDH and B symptoms at diagnosis [26, 62].

## 5. Pathologic Features

### 5.1. Histologic Findings

The histopathological features are frequently ambiguous, thus rendering the correct diagnosis quite difficult. Diagnosis requires a properly evaluated tissue biopsy of mass lesion or lymph node. Excisional biopsy is the gold standard; however, when the site of the disease is difficult to access, core needle biopsy and fine needle aspiration (FNA) may be performed in conjunction with appropriate ancillary techniques for the diagnosis and differential diagnosis. This type of lymphoma is apparently observed more frequently in the immunodeficiency associated cases.

PBL was first described as a specific clinicopathologic entity by Delecluse and colleagues [1] as an aggressive B-cell lymphoma occurring in the oral cavity arising in the context of HIV infection characterized by sheets of plasmablasts without intermingled plasma cells. The presence of a spectrum of plasmacellular differentiation has been introduced in the following years and is a frequent feature of plasmablastic lymphomas outside the oral cavity [63].

The minimum morphological criteria required to diagnose PBL are monomorphic cellular proliferation of plasmablasts, with either centrally or eccentrically placed nuclei with high nuclear-cytoplasmic ratio, a moderate amount of eosinophilic cytoplasm, a high mitotic index, and the absence of neoplastic plasma cells in the background [33, 64].

The article "Plasmablastic Lymphoma: A Review of Current Knowledge and Future Directions" was retracted in 2016. Reasons: plagiarized text; overlap with other authors' work.

Overall, PBL is characterized by cellular proliferation of large atypical cells with immunoblastic, plasmablastic, or plasmacytic features, including eccentric nuclei with a vesicular chromatin, either prominent central nucleolus or peripheral nucleoli, abundant eosinophilic cytoplasm, and a perinuclear hof, in a diffuse sheet-like and cohesive growth pattern (Figure 1). Apoptotic bodies and mitotic figures are frequent, and tingible-body macrophages are easily detectable leading to a starry-sky appearance. Smaller neoplastic cells with obvious plasmacytic differentiation may also be present. Areas of necrosis are occasionally identified [1, 3].

However, these histologic features may be seen in other disorders, such as plasmablastic PCM, BL, DLBCL with plasmacytoid differentiation, PEL, and anaplastic lymphoma kinase- (ALK-) positive DLBCL which make the correct diagnosis challenging [62].

## 6. Immunophenotype

PBL is a high-grade B-cell lymphoma that arises from postgerminal center B-cell. The hallmark immunohistochemical staining pattern of PBL is that of terminally differentiated B-cell. PBL demonstrates little to no expression of leukocyte common antigen (LCA) or the B-cell markers CD20, CD79a, and PAX5. However, the plasma cell markers VS38c, CD38, multiple myeloma oncogene-1 (MUM1), and CD138 (syndecan-1) seem to be almost universally expressed [3, 16, 32]. PBL is characterized by a high proliferation index reflected by Ki67 expression, usually >80% (Figure 2).

Cytoplasmic immunoglobulins are expressed in near 70% of cases. PBL is also variably positive for CD30, epithelial and endothelial markers such EMA and CD31, posing some problems in differential diagnosis with poorly differentiated solid tumors [65]. PBL usually does not express CD56, distinguishing it from true plasma cell neoplasms. Recently, an immunohistochemistry stain for BLIMP1 and XBP1, markers of terminal B-cell differentiation has been proposed to identify PBL; however this finding remains investigational [45] and these markers are often not routinely available.

## 7. Genomic Profile

Currently, very little is known about the molecular genetic basis that drives PBL. One study showed that up to 47% of EBV-positive AIDS-related PBLs are marked by C-MYC translocations, which have previously been associated with other ARLs [55, 64].

*MYC* gene rearrangement is the first recurrent cytogenetic abnormality detected in PBL [55, 62], occurring in approximately 50% of cases. The most common partner for the MYC oncogene is the immunoglobulin gene with translocations most often occurring in the context of complex karyotypes. MYC rearrangements were more often seen in EBV-positive compared to EBV-negative tumors [55].

The article "Plasmablastic Lymphoma: A Review of Current Knowledge and Future Directions" was retracted in 2016. Reasons: plagiarized text; overlap with other authors' work.

Chang et al., studied the genomic profile of 16 cases of PBL, 13 cases of AIDS-related DLBCL, 13 cases of non-AIDS-related DLBCL, and eight cases of PCM [19]. Their findings revealed that the genomic aberration pattern of PBL was more closely related to DLBCL than PCM. These findings suggest that PBL is best classified as a DLBCL based on genomic expression criteria despite the high degree of immunophenotypical similarity between PBL and PCM [19].

In contrast, in a series of four PBL patients showed complex cytogenetic changes that were more closely related to PCM [39]. These findings likely represent the molecularly heterogeneous nature of PBL [6]. Interestingly, two different studies reported single cases showing a concomitant IgH and T cell receptor gene rearrangement [57, 66].

## 8. Differential Diagnosis

The clinical and histopathological features are usually ambiguous, thus rendering the correct diagnosis quite difficult in the absence of an exhaustive integration of clinical, morphological, phenotypic, and molecular features. The diagnosis of such neoplasms could be even more challenging in the setting of extraoral localizations and in immunocompetent patients.

Differential diagnosis with the activated B-cell-like (ABC-like) subgroup of DLBCL and PCM with plasmablastic morphology is still a common problem because of the lack of a distinctive phenotype.

The differential diagnosis includes immunoblastic DLBCL and other lymphoid neoplasms with plasmacytic features such as ALK-positive DLBCL, PEL both classic (body cavity-based) and solid (extracavitary) variants, BL with plasmacytoid differentiation, and plasmablastic plasmacytoma/myeloma (Table 1) [67].

Immunoblastic DLBCL and BL can be excluded on the basis of the characteristic immunophenotypic pattern of PBL with CD20 negativity in combination with positive markers of postgerminal center B-cells and plasma cells, such as CD138/syndecan [1, 9]. CD20 and LCA immunoreactivity is uniformly present with DLBCL and BL and generally absent but may be present in a small proportion of malignant cells in PBL. PBL is distinguished from ALK-positive DLBCL by its lack of expression of the ALK protein, and absence of HHV8 coinfection distinguishes PBL from PEL.

Differentiation from plasmacytoma/myeloma particularly with anaplastic/plasmablastic morphology is the most difficult issue in the differential diagnosis and morphologic distinction is not always possible. In practice, the distinction between PBL and plasmablastic PCM frequently depends on clinical correlation [19]. Detection of paraproteinemia in blood and/or excess light chains (Bence Jones proteins) in urine, lytic bone lesions, and hypercalcemia or anemia favors the diagnosis of PCM over PBL. Immunosuppression, especially HIV-related, is much more frequently associated with PBL as well as the presence of EBV [11]. Of note, PCM and plasmacytoma may occasionally occur in the setting of AIDS [68, 69]. The identification of a* MYC* gene rearrangement can help to distinguish PBL from plasmacytoma as the* MYC* rearrangement is rare in the latter disorder. In addition to lymphoid neoplasms, the diagnosis of PBL can be complicated by its morphologic resemblance to myeloid malignancies particularly extramedullary myeloid tumor which can be excluded by immunohistochemical studies of myeloid markers.

The article "Plasmablastic Lymphoma: A Review of Current Knowledge and Future Directions" was retracted in 2016. Reasons: plagiarized text; overlap with other authors' work.

In brief, although there are wide ranging differential diagnoses, the main differential diagnosis considered is extramedullary plasmablastic myeloma. Though difficult, it is clinically important and critical to differentiate between these two entities, as the treatment for the two diseases is significantly different [19].

## 9. Prognosis

PBL generally has a poor prognosis with most patients dying within 2 years from initial presentation, and long-term survivors are very few. The average survival time reported by Delecluse et al. was a few months, and half of the original 16 patients died within 1 year [1]; however, more recent reports have reported improved survival when treatment with both HAART and appropriate chemotherapy is used, similar to outcomes of HIV-infected patients with other NHLs [21, 22, 40, 70].

Several prognostic factors have been identified in HIV-associated lymphomas. These factors include the International Prognostic Index (IPI) score and CD4^+^ cell count. Data on prognostic factors in PBL are lacking and these analyses are unlikely to be performed prospectively given the rarity of this malignancy [71]. The identification of prognostic factors in this population may allow a better understanding of the biology of this disease.

A large literature review of treated cases of PBL shows an overall response rate (ORR) to chemotherapy of 77%, with 46% of patients achieving a complete response (CR) and 31% a partial response (PR) [72, 73]. Despite a good ORR to chemotherapy, the median OS is 14 months with a 5-year OS rate of 31% [16]. Of note, these survival data represent a variety of therapeutic approaches in a heterogeneous patient population.

However, in a recent literature review, more intensive regimens have not been shown to confer a survival advantage when compared to CHOP/CHOP-like regimens [72, 73].

Patients carrying MYC/IgH gene rearrangement have been shown to have a very poor median OS of only 3 months. The association of MYC with poor prognosis has been suggested by additional studies [55], but based on the small sample size, it should be considered preliminary.

The article "Plasmablastic Lymphoma: A Review of Current Knowledge and Future Directions" was retracted in 2016. Reasons: plagiarized text; overlap with other authors' work.

The use of HAART showed a trend towards statistical significance for a better survival in patients with HIV-associated PBL [73].

It is currently unclear if HIV status alone confers a better prognosis in patients with PBL. In a recent review of the literature, patients with PBL and HIV infection were found to have an OS of 14 months compared to 9 months in HIV-negative patients [26]. A potential explanation for this finding is that the use of HAART may restore immune surveillance to combat the tumor more efficiently. Additionally, other factors, such as extent of disease and performance status, may have also played a role in this difference.

## 10. Therapy

PBL is a therapeutic challenge with a clinical course characterized by a high rate of relapse and death. A standard therapy has not yet been established. Treatment usually consists of chemotherapy with or without consolidation radiation and hematopoietic stem cell transplantation [74]. Various chemotherapy regimens including cyclophosphamide, doxorubicin, vincristine, and prednisone (CHOP), R-CHOP, and cyclophosphamide, vincristine, doxorubicin, high-dose methotrexate/ifosfamide, etoposide, and high-dose cytarabine (CODOX-M/IVAC) are also possible options [73, 75]. Patients with PBL who were not treated with chemotherapy invariably died with a median survival of 3 months [26]. The presence of MYC translocations in a proportion of patients with PBL justifies a more thorough assessment of more intensive regimens.

Due to the lack of CD20 expression, the use of the anti-CD20 monoclonal antibody rituximab is of uncertain utility and unlikely to be of benefit; however it could be considered if partial expression of CD20 is detected within the malignant cells [33]. Although CHOP therapy is often given to treat PBL [16, 23], standard CHOP seems an inadequate treatment [76]. Intensification of induction chemotherapy with autologous hematopoietic stem cell transplantation (auto-HSCT), thought to be a good option in HIV-negative patients with chemosensitive disease, has also been shown to be feasible in HIV+ patients [77, 78].

In the HIV-infected population, the addition of highly active antiretroviral therapy (HAART) also improves prognosis. In a recent study of 70 patients with HIV-positive PBL treated with chemotherapy, the use of HAART was associated with a statistical trend towards improved survival [73]. Interestingly, HAART without chemotherapy has been associated with spontaneous remissions in a few cases [79, 80].

Due to disappointing response and survival rates, the NCCN guidelines recommend against CHOP in favor of more intensive regimens, such as infusional EPOCH, hyper-CVAD, or CODOX-M/IVAC [75]. However, Castillo and colleagues evaluated treatment outcomes in patients receiving CHOP, CHOP-like, and more intense regimens. They reported no statistical difference in the overall survival between the less and more intensive treatment regimens, although only a quarter of the patients reported in the literature have been treated with more intensive regimens than CHOP [73].

The article "Plasmablastic Lymphoma: A Review of Current Knowledge and Future Directions" was retracted in 2016. Reasons: plagiarized text; overlap with other authors' work.

## 11. New Drugs and Future Directions

Due to the rarity of PBL, there is no current consensual standard therapy available. Lack of standard treatment for PBL and its poor therapeutic outcome suggest that new therapeutic approaches are needed. Novel agents used in myeloma therapy are currently applied to PBL considering that PBL shares many morphologic and immunophenotypic characters with plasmablastic myelomas.

One of the newly emerged therapeutic options for PBL is bortezomib, which is a proteasome inhibitor and a cornerstone in myeloma therapy and relapsed or refractory mantle cell lymphoma [81]. Some studies have reported that the proteasome inhibitor bortezomib alone or in combination with chemotherapy may have an antitumor effect in PBL or overcoming the typical chemoresistance of this disease. For the same reason, the use of lenalidomide has been reported in PBL [33]. In recently published cases, bortezomib has shown promising results in PBL [7, 81–85]. Although most of these responses were not sustained, bortezomib represents a new therapeutic option for PBL. Bibas and colleagues have used bortezomib alone or in combination with chemotherapy in patients with PBL and they reported that the results were promising but failed to show any survival advantage over standard chemotherapy [86]. Despite initial promising results, the drugs were used at case report level and the response with the new agents was transient and should be further explored in larger clinical trials [7, 86, 87].

Owing to improved gene transfer technology, novel adoptive cellular therapies have been developed. Adoptive transfer of tumor-reactive T cells into cancer patients with the intent of inducing a cytotoxic antitumor effector response and durable immunity has long been proposed as a novel therapy for a broad range of malignancies [88, 89] The introduction of genes, adoptive cellular therapy, involves the encoding of artificial receptors known as chimeric antigen receptors (CARs). These CARs are recombinant receptors that comprise an extracellular antigen-targeting domain in conjunction with one or more intracellular T cell signaling domains that can be introduced into T cells by genetic modification to redirect the specificity and function of immune effectors. CAR-modified T cells targeted to the B-cell-specific CD19 antigen have demonstrated promising results in multiple early clinical trials, supporting further investigation in patients with B-cell cancers. Recent preclinical studies support additional genetic modifications of CAR-modified T cells to achieve optimal clinical efficacy using this novel adoptive cellular therapy. However, its use had limited clinical application in the treatment of hematological malignancies. This approach is further limited by complications including a lack of efficient cloned TCR expression [90]. An ongoing study is evaluating the therapeutic value of autologous EBV-specific CAR T cells with CD30 as the target. Potentially, CAR T cells can be directed against EBV antigens in patients with EBV-associated lymphomas including PBL [23].

The article "Plasmablastic Lymphoma: A Review of Current Knowledge and Future Directions" was retracted in 2016. Reasons: plagiarized text; overlap with other authors' work.

As reported before approximately 30% of PBL cases express the activation marker CD30 [32, 55] and a recent report showed response to brentuximab vedotin in a patient with CD30-expressing relapsed PBL [91]. More recently, a case series of 3 previously untreated patients with PBL, 2 of them HIV-positive, has shown efficacy with the combination of bortezomib and dose-adjusted EPOCH [92].

## 12. CNS Prophylaxis

Considering the high risk of progression during the treatment or recurrence during the remission, the use of intrathecal prophylaxis is considered a mandatory part of the systemic treatment [93]. Controlled studies on this field are not available, so the standard procedure has not been defined. However, intrathecal methotrexate or cytarabine are administered at each cycle of chemotherapy, based upon institutional preference [94].

## 13. Refractory or Relapsed Patients

Treatment in patients with refractory or relapsed HIV-associated PBL is considered palliative although some cases of long-term survival have been described. In general, a more intensive chemotherapy is planned for relapsed patients, and for fit patients intensification of chemotherapy with autologous HSCT may be an option [33].

As the outcome of patients with relapsed or refractory PBL is very poor [73] and the outcome is significantly superior in patients with relapsed NHL who received autologous HSCT compared with those who did not, it seems rational to explore the use of autologous HSCT earlier in the course of disease: at least in the patients with high-risk disease to improve the overall survival (OS) rate [93]. Due to the dismal outcome of salvage chemotherapy, autologous HSCT appears to be feasible and possibly beneficial compared with multiagent chemotherapy in the setting of relapsed and refractory disease [77, 95]. Effectiveness of such therapy was not significantly different between HIV-positive and HIV-negative patients, in terms of treatment-related mortality, opportunistic infections, immune recovery, and OS; however, allogeneic BMT is a more limited option in HIV-positive relapsed PBL [77, 78].

The article "Plasmablastic Lymphoma: A Review of Current Knowledge and Future Directions" was retracted in 2016. Reasons: plagiarized text; overlap with other authors' work.

## 14. Conclusion

PBL has a predilection for immunocompromised individuals based on its prevalence in both HIV-positive patients and in those undergoing solid organ transplantation. PBL is best classified as a form of DLBCL. However, based on immunohistochemical data, PBL is much more similar to PCM. Clinically, it has a predilection for oral cavity involvement, a feature not typically seen in other lymphoid malignancies. Recent studies have shown a high prevalence of MYC translocations that may contribute to its aggressive nature. The pathogenesis has not clearly been defined but is thought to involve dysregulation of terminal B-cell differentiation and apoptosis, potentially via the effects of MYC translocation and EBV infection. Treatment has been centered on CHOP chemotherapy with good response, but poor survival; however, more intensive therapies are recommended. Recent case reports of a good clinical response to bortezomib are encouraging and may provide clues to the underlying pathophysiology of PBL. Finally, it is worthwhile to highlight that no prospective therapeutic trials have been done specifically in patients with PBL.

## Figures and Tables

**Figure 1:** Histopathologic features of PBL: (a) H&E stain shows sheets of large atypical lymphoid cells with plasmacytic differentiation with abundant cytoplasm, paranuclear hof, and large nuclei; (b) it displays large cells with an immunoblastic appearance, with central oval nuclei with prominent nucleoli and moderately abundant cytoplasm.

**Figure 2:** Selected immunophenotype of PBL: the PBL cells demonstrate immunoreactivity to CD138 (a), lambda light chain,* ISH* (b), and HHV8 (c) and negativity for CD20 (d) and CD56 (e). Proliferation index is high (f).

**Table 1:** The main differential diagnosis of PBL.

Clinical presentation	Frequently oral cavity	Often extranodal (jaws and orbits)	Wide variety of presentations	Involves body cavity	Wide variety of presentations	BM (extramedullary in plasmacytoma)	BM (extramedullary in plasmacytoma)
Immunocompetency	+/−	++	+++	+/−	+	++	++

Association with HIV	+++	++	++	+++	−	−	−

Association with HHV8	+/− (usually −)	−	−	+	−	−	−

LCA	+/−	+	+	+/−	+/−	+/−	+/−

B-cell markers							
CD20	−	+	+	+/−	−	−	−
CD79a	+/− (usually −)	+	+	−	−	+/− (usually −)	+/− (usually −)

CD138	+	−	−	+	−	+	+
CD56	+/− (usually −)	Rare +	Rare +	Rare +	+/−	Usually +	Usually +

Ki67	High >70%	High >90%	High <90%	High >80%	High >80%	Low	High >70%

Other	BLIMP1+	CD10 +	BCL-6 Usually +	CD30 Usually +	ALK+	Serum M-spike CRAB	Serum M-spike CRAB

CRAB: hypercalcemia, kidney disease, anemia, and bone lytic lesions [67].
